# The Collection and Utilization of Web Resources for Teaching World History Based on Data Mining Technology

**DOI:** 10.1155/2022/9124952

**Published:** 2022-08-01

**Authors:** Xia Wu

**Affiliations:** School of History Culture and Tourism of Liaocheng University, Liaocheng 252000, China

## Abstract

The foundation of research for academics involved in world history education and research is timely access to pertinent foreign information, comprehension of domestic and international academic developments, and access to fundamental historical materials and research outputs from our ancestors. As a result, it is essential to investigate the necessity and viability of using network resources on the basis of analysis in order to respond to the educational philosophy of the new curriculum reform and adapt to the development of modern teaching methods based on network technology. The creation and use of curriculum resources is an essential component of curriculum development and a crucial assurance for curriculum implementation. The growth and acceptance of online learning will undoubtedly influence how history education is practised around the world. The scarcity of online learning resources is currently a bottleneck impeding the growth of online education. On the other hand, data mining (DM) takes the massive amount of incomplete data and extracts the useful knowledge and information hidden within it. This paper explores the “DM” process of utilizing online resources and suggests a method for gathering and utilizing world history education online resources based on DM technology. The experimental results show that the test interval between MapReduce and DM gradually increases with the increase of data volume. The advantage of DM is more obvious, as the average test time of DM is 27.66 seconds shorter than that of MapReduce. Therefore, DM has high application value in the field of search engines and social network analysis.

## 1. Introduction

The philosophy and approaches to teaching world history have significantly changed in the modern era as the Internet becomes more and more integrated into people's daily lives [1]. All facets of society have been profoundly impacted by the advancement and use of modern science and technology, with computer networks and multimedia technology serving as its core [2]. The education sector also adopts the modern trend of Internet integration [3]. The use of a large number of online course resources in education has had a profound effect on the field of education [4]. Schools in various parts of China have accelerated the development of network hardware and actively promoted online education in response to the development trend of information technology and networking [5]. Theoretical studies on online teaching have recently surfaced as the subject has recently gained popularity in the education sector. However, improvements in the world history curriculum have been made in terms of teaching resources, course content, teaching methods, and pedagogy as a result of the complex and diverse Internet environment. However, it also encounters a number of difficulties and issues, including an abundance of information, uneven information quality, violence, and vulgarity.

The web has developed into a vital source and archive of knowledge for people in their daily work and study today. Participants can access services in various languages, such as daily information advice, meeting arrangements, emergency services, and taxi hailing services. People demand tools that can be used to filter information and get rid of information bubbles, hard shells, and useless packaging because they are faced with an infinite variety of information. The use of the Internet, its expansion, and how to access its information have all become difficult. DM was created in such an environment. The characteristics of complex data and extensive network resources, however, make DM work challenging.

DM, also known as knowledge discovery in databases, is a hot topic in artificial intelligence and database research. By DM, we mean the process of implicitly revealing previously unknown and potentially valuable information from a large amount of data in a database. DM consists of three steps: data preparation, regular discovery, and regular expressions. For world history teachers, this new and convenient tool is an indispensable tool to support educational and scientific research. With the development of web technology, the abundance of web resources continues to explode. In response to the desire to discover knowledge from data, there are many distinguished researchers in various fields such as databases, pattern recognition [6–8], machine learning [9–11], artificial intelligence [12, 13], statistics, visualization [14, 15], and parallel computing. The innovation points of this paper are as follows:

1. Combining network resource collection and DM technology, combining learner physical and mental characteristics, investigating some workable resource collection algorithms based on DM technology, changing the conventional brainwashing method, and technicalizing the learner's world history education situation are some examples of these approaches.
2. Based on the previous research, we keep analyzing the application of DM technology in teaching the collection and utilization of web resources, that is, analyzing the basic process of DM in teaching web resources and proposing the ways of resource utilization based on DM technology.
3. Improved parallelization of DM to create a networked world history learning environment is analyzed. The resource collection algorithm based on DM technology is always able to provide a democratic and free way of learning and communication for world history students and world history enthusiasts.

## 2. Related Work

### 2.1. Collection and Utilization of Network Resources

All types of data are being generated in significant amounts as society transitions into the era of network information. These data conceal a wealth of significant information, and it is becoming increasingly important to identify specific patterns and insightful information within them. Users can interact with keywords, receive summaries of related keywords on DM, sort related keywords by relevance, and highlight related keywords. A good resource collection mechanism should take into account elements such as collection latency, topology, network, resource hit ratio, fault tolerance, and scalability because resource collection algorithms are also very diverse.

Singh and Yassine reviewed the evolutionary path of online teaching and learning, analyzed the problems of online teaching and learning with relevant data, and discussed four aspects of effective online teaching and learning pedagogical theory exploration, model construction, practical research, and faculty evaluation [16]. Long discussed the effectiveness of online course training. The use of online resources in world history pedagogy was studied by drawing on new teaching methods using computers as tools: modern teaching methods such as teaching based on online resources, multimedia technology, and network technology [17]. Li describes the methods and ideas for the development, editing, and management of each course learning module in relation to the theoretical and practical development stages of online course architecture [18]. Rahman et al. argue that teaching world history courses using online resources is not a traditional teaching method, nor is it a way to support or teach computers in multimedia classrooms [19]. According to Zeng, web-based course resources are information technology aspects. A new form of development of curriculum resources refers to the use of computer systems to disseminate and manage curriculum resources through communication devices and network software [20].

The volume of various information amounts to hundreds of millions, which not only provides material security for us to use network resources for education and research but also makes the access and utilization of network resource an essential skill.

### 2.2. DM Technology

With the rapid development of the Internet, the massive information storage, convenient transmission, and interactive features that transcend time and space have greatly changed people's lifestyles. The unlimited Internet resources provide teachers with rich educational resources on the one hand and satisfy students' curiosity on the other. Faced with the challenge of “abundant data and lack of knowledge,” we urgently need powerful data analysis tools that can discover useful knowledge, relationships, and rules in the complex and huge data, thus bringing great value.

For large data sets, Grdinaru et al. first sorted the original data set, analyzed the virtual memory implementation mechanism of the operating system, and optimized the original algorithm in terms of the spatial and temporal locality to become an input-based algorithm output aware mining algorithm [21]. Huizhen can solve this problem to a large extent by using high-performance computers and parallel computing. This is because parallel computing can provide the computational power needed to process large amounts of data, and clusters can be used to increase the computational power as the data grows [22]. Wei et al. studied the hardware and software infrastructure for distributed association rule mining algorithms. They considered distributed DM including distributed mining algorithms, parallel mining algorithms, distributed parallel databases, and other research [23]. Terbusheva proposed that resource management systems and network management systems data are acquired with certain correlations, including horizontal and vertical correlations [24]. Slater et al. statistically sampled the original data set and clustered the sampled small data set with similar algorithms including random sampling K-means [25].

DM can also be classified according to applications, including the financial industry, stock market, and so on, which have their own applicable and widely adopted DM methods. As an emerging technology, the development of DM must also follow the general trend of technological development. How to use DM technology to obtain knowledge from these big data sets has become an important research area.

## 3. Thoughts on Collection and Utilization of Teaching Network Resources Based on DM Technology

### 3.1. Resource Collection Algorithm Based on DM Technology

The resource collection algorithm is built on the topology of the network, and the corresponding resource collection algorithm is designed according to the network topology [26]. In terms of dynamic scaling, the computational power of the resource collection algorithm supports dynamic scaling, and the user can expand the computational power on demand [27]. If the comparative analysis of factor data with different magnitudes is to be performed simultaneously, they need to be normalized. The value of *i* factor *j* in all samples is

(1) $$\begin{array}{c} Z_{i,j}=\frac{X_{i,j}-\mu_{j}}{\sigma_{j}}, \end{array}$$

where *μ*_*j*_– mean value of *i*-th factor and *σ*_*j*_– the standard deviation of *j*-th factor.

The main workflow of the current resource collection can be roughly divided into the process of establishing the index and the user collection process, as shown in Figure 1.

First, the initiating node sends a query request to all its neighbouring nodes by means of a broadcast, which in turn broadcasts it to its own neighbouring nodes. The DM technique is application-oriented from the beginning. The error is propagated in the reverse direction by continuously updating the weights and the bias that expresses the network prediction error. The error is calculated as follows:

(2) $$\begin{array}{c} {\text{Err}}_{j}=O_{j}\left(1-O_{j}\right)\left(T_{j}-O_{j}\right), \end{array}$$

where *j*– output layer nodes, Err_*j*_– error, *O*_*j*_– actual output, and *T*_*j*_– a known target value based on a given training sample.

It goes beyond simple search query calls against specific databases to perform micro- and macrostatistics, analysis, synthesis, and reasoning on this data. To guide the solution of real-world problems, find correlations between events and even use existing data to guide future activities. There are also links to a dozen other specialized online virtual libraries of world history belonging to different institutions, such as the Google Rankings Virtual Library for Pacific historical research and the Virtual Library for economic and business history [28]. Logically dividing the database into several separate blocks, one block at a time is considered individually, and all frequency sets are created for it; then the generated frequency sets are combined to create all possible frequency sets; and finally, these computational sets are supported. Detect the existence of solutions within the initial solution set  *T*  that meet the requirements of the flexibility constraint. If it exists, it is marked as a feasible solution; otherwise, the parameter range of the constraint index interval is adjusted until a feasible solution exists; assuming that *B* is a diagonal matrix, the above equation can be transformed into the following form:

(3) $$\begin{array}{c} e\left(y,z\right)={\left[\sum_{j=1}^{p}b_{\text{ij}}{\left|y_{j}-z_{j}\right|}^{s}\right]}^{1/2}, \end{array}$$

where *b*_ij_– the *i*, *j* data attribute in the database.

Since high-frequency and closed item sets are much smaller than frequent item sets, using a closed item set grid can reduce the search space and the number of scans in the data set.

Secondly, it can selectively forward to a subset of adjacent nodes to reduce the number of visited nodes, reduce redundant messages in the network, and save network bandwidth. Since electric load data are cyclical, a small period of 24 hours should be used to clean up the world historical load data, and the mean substitution method should be used to mine the load data:

(4) $$\begin{array}{c} \bar{A}\left(d,t\right)=\frac{1}{n}\sum_{d=1}^{n}A\left(d,t\right), \end{array}$$

where $\bar{A}\left(d,t\right)$– average value of load value.

The staff reviews the information and then manually compiles a summary of the information before categorizing it into predefined categories [29]. Directory collection engines are collections that collect website information manually or semiautomatically. The client sends data to all data copies after obtaining write access, and once all data copies have received the updated data, the client sends a write request control signal. The system can be broken down into three layers based on the relationships between the frameworks because the client uses various frameworks to carry out various functions. The architecture is shown in Figure 2.

The accuracy of the algorithm is guaranteed at least by all possible frequencies set in a particular block. Data decomposition overcomes memory bottlenecks and improves the efficiency of mining large data sets by reading a portion of the segmented block data into memory, processing it, and finally merging the entire processing result. Root-mean-square error is used to measure the deviation between the predicted and true values by reflecting the degree of variance in the data set:

(5) $$\begin{array}{c} \text{RMSE}=\sqrt{\frac{\sum_{i=1}^{n}\left(\sigma_{i}-\overset{↔}{\sigma_{i}}\right)}{n}},\;i=1,2,\ldots ,n, \end{array}$$

where $\overset{↔}{\sigma_{i}}$– a predicted value in the set of prediction results, *σ*_*i*_– corresponding actual load value, and *n*– number of predicted values in the set of prediction results.

Finally, the process is terminated when the query results are satisfied or the maximum depth limit is reached. In flooding, the number of nodes grows exponentially with increasing depth [30]. Due to a large amount of information in the network itself, it will undoubtedly expand the educational resources like never before. Therefore, data management in cloud systems tends to use the data management model of columnar storage in the database domain. However, these small data blocks contain only a small fraction of the information in the original large data set, and only a set of local frequency terms are found. Therefore, when users search and collect resources using collection engines, they select the most suitable collection engine for their goals and choose collection strategies and collection techniques that reduce the size of the transaction set used for future scanning. A basic principle is that when a transaction does not contain a large item set of length *k*, it must not contain a large item set of length *k*+1.

### 3.2. Ways of Resource Utilization Based on DM Technology

Examining the current state of online resources—that is, the need to use them—is the first step in determining how they relate to world history education. In order to make it happen, the ultimate goal of creating online educational resources is to offer online education, support students' independent learning on the Internet, assist teachers in organizing online educational materials, and make it possible for educational administrators to monitor and assess educational effectiveness. Therefore, the ability to manage large data sets effectively requires data management skills. Create that data model pipeline using DM to extract random, enormous, and incomplete real-world application data as objects. The flow of DM is shown in Figure 3.

First of all, we should give full play to the role of network technology and integrate educational resources. By integrating teaching resources, we can save the time of explaining and boarding and focus our time and energy on the breakthrough of specialties and difficulties. Constructivism also emphasizes that the teacher is both a helper and a guide to help students learn knowledge. The lecture process should take into account the cognitive background and knowledge base of the students and help them construct a knowledge system that focuses on the BER and reliability of service time correlation. Given a transaction database with a user input with minimum support *w* min Sup, if the t attribute set *X* is frequent, then its support number and minimum support number should satisfy, respectively:

(6) $$\begin{array}{c} \text{SC}\left(X\right)\geq \frac{w\text{ min Sup}\times T}{\text{MAX}\left(w_{i}\right)}, \end{array}$$

(7) $$\begin{array}{c} B\left(X\right)=\left[\frac{w\text{ MAX}\left(w_{i}\right)\min\text{ Sup}\times T}{\text{MAX}\left(w_{i}\right)}\right]. \end{array}$$

These conditional patterns are then mined separately. When the amount of raw data is large, it can also be combined with a partitioning approach so that an FP-Tree can be placed in the main memory. The level-weighted support of the item set *X*={*i*_1_,  *i*_2_,…, *i*_*k*_} is defined as follows:

(8) $$\begin{array}{c} {\text{Sup}}_{h}=\text{max}\left\{h_{1},h_{2},\ldots ,h_{k}\right\}\times \text{Sup}\left(X\right), \end{array}$$

where Sup(*X*) is traditional support count of item *X* and Max{ *h*_1_, *h*_2_,…,*h*_*k*_} is weight of items.

The BER of the service is somewhat time-dependent, and typically, the consequences of the long-term presence of BER are more severe than the instantaneous BER problem. Therefore, these local candidate frequent item sets generally need to be written to disk, freeing up memory space for frequent item set discovery for the next data block. The weight of item set *X*={*i*_1_, *i*_2_,…, *i*_*k*_} is given as *w*_*j*_, where 0 ≤ *w*_*j*_ ≤ 1,  *j*={1,2,…, *k*}. The weighted support of item set *X* is

(9) $$\begin{array}{c} W\text{ Sup}\left(X\right)=W\left(X\right)\times \frac{\text{Sup}\left(X\right)}{T}, \end{array}$$

where *W*(*X*)– Max{*w*_1_, *w*_2_,…, *w*_*k*_}.*T*– total number of transactions in the database.

Second, the creation and use of PPT courseware can help teachers effectively integrate and present world history online course resources to optimize the teaching process and achieve good teaching results. This is because online resources tell students that learning is interactive learning, emphasizing discovery and creative learning as well as the learning process. When all data blocks have been processed, the original large data set must be rescanned, a set of candidate frequency items on disk must be computed, and the true global set of frequency items must be selected. The maintenance and analysis of the network service life cycle are performed mainly for each cycle of the service, and the system has to estimate the BER of the network service and maintain the BER detection values. Combining the idea of weight set with maximum weights of horizontal weighting with vertical weighting, for the item set *X*={*i*, *i*_2_, *i*_3_,…, *i*_*a*_}, the mixed weighted support of *X* is defined as follows:

(10) $$\begin{array}{c} {\text{Support}}_{m}\left(X\right)=h_{x}\;{\text{sup}}_{v}\left(X\right)=\text{max}\left\{h_{1},h_{2},\ldots ,h_{k}\right\}\frac{\sum_{i=1}^{n}\left(V_{i}\text{ Count}\left(X_{i}\right)\right)}{N_{v}}. \end{array}$$

Finally, to enhance the effectiveness of classroom instruction and to take advantage of microlesson resources that support world history education and encourage reflection, students can watch and study microlessons online to prepare for class or to consolidate and reinforce their knowledge. Big data from web resources are structured, and using SQL statements to query it at random can cause issues with data computation performance, necessitating the use of a new query method. The original data set is scanned twice, and a large number of candidate frequency items are written and read, so the partition-based method still needs more I/S. Large data sets must be managed effectively, and specific data must be found in very large data sets. Task-related data, knowledge primitives for primitive mining, background knowledge primitives, and interest measurement primitives are the five main definitions of DM primitives in DM Query Language (DMQL).

## 4. Application Analysis of DM Technology in the Collection and Utilization of Teaching Network Resources

### 4.1. Analysis of the Basic Process of DM in Network Resources

Web resources are an integrated system of hypertext and hypermedia constructed by combining computer technology and communication technology. The current web resources are very rich, including general historical and disciplinary knowledge, universal knowledge and specialized research information. Therefore, the first thing to do before doing DM is to define the problem, clarify the problem and target tasks, and determine the purpose of DM. Build the simulation model on the platform and run the experiment under the same conditions. The experimental results of comparing the number of messages generated by flood traversal of all nodes in the FIFSM model and DM are shown in Figure 4.

First, it contains noise; contains incomplete, ambiguous, real-world application data with high randomness; and performs large-scale cleaning of data, denoising, deriving calculations to fill in defects and incomplete data, correcting anomalous data, and removing redundant data. Large data sets cannot be fully read into memory for processing, and the mapping of large data sets may exceed the available system memory and cannot be fully constructed in memory. In this case, the rating matrix is very sparse, and the situation where the similarity becomes zero is called neighbour transmission loss because there are two similar users but few common rating entries. Therefore, during the mining process, a way is needed to save some of the data to disk, freeing up more memory space for subsequent data. The manually initialized uniform resource locator has a high probability of topic relevance within a certain link distance. It is also used in conjunction with web filtering techniques, which first crawl web pages using a breadth-first strategy and then filter out irrelevant pages. The acceleration ratio is the ratio of the time required for the same task to run on a uniprocessor system and a parallel processor system.  Table 1 shows the DM tests for 15,000 records on clusters with different numbers of nodes, where the amount of data is the same and the level of support is also the same.

Secondly, data from different sources, formats, characteristics, and attributes must be collected physically or logically in order to prepare for the subsequent set of data processing. According to the model definition and description to make the DM system regular, various DM systems can share the model, and the DM model can be nested in the middle of the application system for the purpose. The breadth-first collection traversal is similar to the hierarchical traversal of a tree, and the traversal process can be described simply. In terms of accessing information and sharing information resources on the web, students only need to master key computing skills such as how to browse the web, use DM, and understand and learn how to download materials. Then they can independently access a variety of different sociocultural information, educational reference information, advanced technological information, and so on. In the FIFSM flooding algorithm, the query message propagates the forwarding interval of the receiving node, and the loss of the query message leads to the loss of the nodes in the forwarding interval. The percentage of duplicate messages flooded to all nodes is shown in Figure 5.

Finally, in the DM step, the appropriate algorithm should be selected based on the nature of the data itself and the expected ability to extract the implied patterns from the data. Complex DM operations consisting of multiple data sources and DM modules require the exchange of results between different modules. The main components of the Predictive Model Markup Language (PMML)have this flexible model exchange capability and data format conversion, enabling the separation of the model from the data and tool components. If there is a solution, Stormline collection always finds the best solution, but from some point of view, depth-first is faster and Stormline has to traverse every node, so it takes a lot of time.

### 4.2. Parallelization Improvement Analysis of DM

Algorithms exist for DM to reduce the complexity of prediction scores, but this reduction is negligible in the face of large amounts of data. In the collection process, the best priority collection strategy calculates the predicted candidate URLs based on the similarity to the target or relevance to the topic according to the web analytics algorithm. Therefore, the parallelization improvement of the “desired” pages by DM through the threshold web analysis algorithm is the locally optimal collection algorithm. It is generally used as a transport layer protocol to ensure the reliability of message transmission and to prevent message loss due to link failure, and the node failure rate of 10 and 20 is shown in Figure 6.

Firstly, in the early stage of data sorting, the messy data can be sorted by user ID to select unnecessary information and speed up the later data processing. The hypothetical and complex nature of web information determines that world history teachers and students face very rich information of web resources, and screening the real and valid resource information is an important step. The central goal of each cluster is this kind of data. It calculates the average value of records, calculates the size of each data record from its central object, and then subdivides that data record according to its minimum distance. The use of IO devices is inevitable, but the input data depends. As for the file blocks allocated by the platform file system, each node processes only its own allocated file blocks and does not compete with each other for resources, but the heuristic collection gives some distribution predictions. With the help of specific knowledge, it is possible to obtain information resources that can be directed to approximately the collection. To evaluate the success rate of the mechanism DM in a dynamic environment, the experiments set the working period to 30 seconds and the flood count to 15, 30, and 45 and show the node hit rate results. The results are in Figure 7.

Second, computing user similarity is a continuous concept that computes the cosine or Pearson values between two users in turn. It is not suitable for finding classes with large size differences or classes that exhibit nonconvex shapes and are sensitive to noise and anomalous data. Even if the amount of such data is small, it is not effective for clustering. It is important to note that the class should not be turned into a demonstration class and that the teaching method should not be used from the beginning to the end with Internet resources and computers and multimedia. Points and difficulties. In the case of DM, the efficiency of the algorithm is verified by node comparison.  Table 2 shows the amount of data and time used for testing.

The test interval between MapReduce and DM gradually increases as the amount of data increases. The advantage of DM is even more pronounced, as the average test time for DM is 27.66 seconds shorter than MapReduce. As DM progressively builds the best solution, each step makes the best decision based on specific criteria. Once a decision is made, it cannot be changed. Most operations can be seen as grouping and merging of collection elements, making them well suited for parallelization using the programming model. When a node leaves, it may create empty routing entries on other nodes, but the number of nodes in each entry can reach the maximum node redundancy. Assume a redundant node count of 0–40, a duty cycle of 60 seconds, and a node count of 15.  Figure 8 shows the control message count curve for DM.

Finally, whenever a query is made to the nearest neighbour set or a neighbour evaluates a piece of data, it first checks to see if the record already exists in memory; if not, it reads the file to get the record and then puts the record into memory. A wide range of educational information is available to students thanks to the informational diversity of web resources. In order to choose the information that is relevant to students' cognitive structures and appropriate for a student production, teachers should be cautious when choosing web resources. The validity and applicability of the patterns discovered by DM have been evaluated using a number of different techniques. It searches for patterns that represent knowledge and are genuinely valuable based on a particular metric of interest. The length of each operation's set of transaction items affects how much space is required. This is due to the fact that following each transaction between a set of transaction items, it creates space to store that set of transactions in that set of items, checks to see if the length of that set of transactions satisfies the support, concludes, and then creates space.

## 5. Conclusions

With the advent of the Internet era, Internet resources are applied to world history education as an integral part of the new curriculum resources proposed by the new curriculum reform. The use of Internet information media to develop and utilize world history curriculum resources is both a general trend and a requirement of the new curriculum. In order to make full use of this valuable resource, we must be familiar with various academic information sources, frequently explore various databases and their deployment and access, and build our own essential teaching databases. The rapid development of DM technology has been made possible by the vast amount of data resources the world possesses today and the great need to transform these data resources into information and knowledge resources. Starting from the teaching practice of world history courses, this paper combines theory and practice to define and describe web resources using DM technology and to fully explore and analyze the resources based on DM skills in world history courses using web resources. Therefore, the method of collecting and utilising the network resources of world history education based on DM technology is used to update and utilize various digital academic information in a timely manner and to take advantage of the advantages of network technology to continuously improve and perfect teaching and learning.

## Figures and Tables

**Figure 1:** Index building process and user collection process.

**Figure 2:** Client-side three-tier architecture.

**Figure 3:** Process of DM.

**Figure 4:** Number of messages flooding through all nodes.

**Figure 5:** Percentage of redundant messages flooding through all nodes.

**Figure 6:** Node loss rate of flooding under link failure.

**Figure 7:** Hit rate of nodes in a dynamic environment.

**Figure 8:** DM control message number curve.

**Table 1:** Tests under different nodes.

Number of nodes	Elapsed time (s)	Speed-up ratio
33	342	3.293
78	527	4.186
125	673	6.334

**Table 2:** Test data and time.

Number of records	Map reduce test time (s)	Data mining (s)
50	45.26	23.21
100	56.87	28.78
150	67.23	34.38
Average test time	56.45	28.79

## Data Availability

The data used to support the findings of this study are available from the author upon request.
